# Blockchain-IoT-Driven Nursing Workforce Planning for Effective Long-Term Care Management in Nursing Homes

**DOI:** 10.1155/2021/9974059

**Published:** 2021-11-12

**Authors:** Y. P. Tsang, C. H. Wu, Polly P. L. Leung, W. H. Ip, W. K. Ching

**Affiliations:** ^1^Department of Industrial and Systems Engineering, The Hong Kong Polytechnic University, Kowloon, Hong Kong; ^2^Department of Supply Chain and Information Management, The Hang Seng University of Hong Kong, Shatin, Hong Kong; ^3^Department of Mechanical Engineering, University of Saskatchewan, Saskatoon, Canada; ^4^Department of Mathematics, The University of Hong Kong, Pok Fu Lam, Hong Kong

## Abstract

Due to the global ageing population, the increasing demand for long-term care services for the elderly has directed considerable attention towards the renovation of nursing homes. Although nursing homes play an essential role within residential elderly care, professional shortages have created serious pressure on the elderly service sector. Effective workforce planning is vital for improving the efficacy and workload balance of existing nursing staff in today's complex and volatile long-term care service market. Currently, there is lack of an integrated solution to monitor care services and determine the optimal nursing staffing strategy in nursing homes. This study addresses the above challenge through the formulation of nursing staffing optimisation under the blockchain-internet of things (BIoT) environment. Embedding a blockchain into IoT establishes the long-term care platform for the elderly and care workers, thereby decentralising long-term care information in the nursing home network to achieve effective care service monitoring. Moreover, such information is further utilised to optimise nursing staffing by using a genetic algorithm. A case study of a Hong Kong nursing home was conducted to illustrate the effectiveness of the proposed system. We found that the total monthly staffing cost after using the proposed model was significantly lower than the existing practice with a change of −13.48%, which considers the use of heterogeneous workforce and temporary staff. Besides, the care monitoring and staffing flexibility are further enhanced, in which the concept of skill substitution is integrated in nursing staffing optimisation.

## 1. Introduction

The percentage of the elderly population (i.e., those aged 65 or above) in almost every developed region is growing at a significantly faster rate than any other age group due to declining fertility rates and longer life expectancies [1]. As essential facilities in the geriatric care management, nursing homes worldwide are experiencing severe shortages of nursing staff, along with higher service demands which are only expected to further increase in the near future [2]. While the ageing population trend has pushed the development of long-term care services and facilities and despite nursing homes being an essential component of the healthcare industry, this issue has received limited attention in academia. Firstly, elder residents in nursing homes have diverse and unique service profiles, which are used to formulate customised care plans by doctors, nursing staff, and social workers. Secondly, the elderly's health deteriorates over time, resulting in the dynamicity of their requirements and appropriateness of care services—and therefore the demand for healthcare resources—relatively fluctuating. Hence, maintaining a sufficient service capacity in terms of frontline nursing staff is a consistent challenge in healthcare management. Due to the complexity and volatility of today's working environment, effective nursing workforce planning is as important as it is challenging for nursing homes. Employing effective nursing staffing optimisation is regarded as a promising method to enhance service capacity, provide high quality service at a low operational cost, and maintain a staff workload balance [3, 4]. However, further to typical optimisation problems, nursing staffing optimisation considers the continuous changes and customisations of residents' requirements, thereby necessitating the regular updating of optimal staffing solutions. In so doing, reliable and secure data acquisition from elderly residents is essential to facilitate staffing optimisation in nursing homes. As shown in Figure 1, the elderly has their own customised care plans upon their admission to nursing homes. These plans include the specifications, requirements, and customised services to maximise the quality of care (QoC) of the nursing services. These individual needs are combined in the ward-level to generate a set of requirements and customisations for the nursing care provided.

These are then consolidated at the nursing home level, thus showcasing how optimised nursing staff demand planning is essential for allocating an appropriate level of work to satisfy requirements and customisations at the lowest costs. Since the care plans, requirements, and service customisations are not fixed to the elderly, controlling and monitoring care services throughout the whole nursing home is challenging task. In this study, the blockchain-IoT-driven healthcare service devices are exploited to effectively control and monitor individual care services, where the blockchain is applied to establish secure data acquisition and reliable service records of the elderly [5]. IoT is deemed to be robust to interconnect physical objects, including human being, into a digital platform by using various sensors, actuators, and machines, so as to formulate intelligent applications [6]. Incorporating blockchain in IoT, namely, blockchain-IoT, can leverage the benefits of blockchain technology to strengthen system security and privacy preservation [7]. More importantly, the trust on data and system process can be established and spread in the peer-to-peer network. Based on the collected data via the blockchain-IoT-driven platform, the nursing staffing optimisation was designed to consider previously unaddressed factors, such as staff-task flexibility and heterogeneous workforces, which largely impact nursing staff planning. The platform seeks to manage nursing staff in a cost-effective manner, while concurrently reasonably allocating tasks among all available nursing staff. More importantly, the concept of nursing staff “skills”—classified into managerial and professional aspects—was incorporated into the above model. Therefore, the proposed nursing staffing optimisation can more specifically allocate and balance workloads, thereby resulting in effective geriatric care management.

The next section will review the relevant literature on blockchain, the IoT, and nursing workforce management in care services. The formulation of the proposed blockchain-IoT-driven system is presented in Section 3.  Section 4 provides the algorithm designed to solve the nursing staff optimisation problem. A case study of a nursing home in Hong Kong is presented to illustrate the effectiveness of the proposed system and model, and its results are discussed in Section 5. Finally, conclusions and recommendations for future research are summarised in Section 6.

## 2. Literature Review

In this section, a literature review will synthesise (i) blockchain and the IoT in long-term care services, (ii) factors affecting nursing workforce planning in nursing care services, and (iii) existing approaches for staffing optimisation.

### 2.1. Blockchain and the IoT in Long-Term Care Services

The IoT, which is generally defined as the interconnection between physical objects (or “things”) and the digital world over the Internet, has been actively investigated in the context of healthcare management [8]. To be more specific to medical and healthcare scenarios, the Internet of medical things (IoMT) and the Internet of healthcare things (IoHT) are two emerging paradigms specialising on smart health [9]. All healthcare information can be appropriately considered so as to improve patient decisions and treatment effectiveness, which can be further extended to long-term care services. Tang et al. [2] adopted the IoMT technology to collect several biometric data, including blood pressure, heart rate, oxygen saturation level, body temperature, and blood-glucose level, via wearables, thermometers, and glucometers. All the collected data are used to support the decision-making process in the formulation of individual care plans (ICPs). Asif-Ur-Rahman et al. [10] explored a heterogeneous framework for IoHT, comprised of mist, fog, and cloud computing to structure the data transmission and processing for healthcare applications. While the value of the IoT to the healthcare industry has been persuasively showcased, academics and industrial practitioners have raised concerns over system vulnerability and cybersecurity. Blockchains are regarded as promising tools to enhance security and privacy in healthcare data management, in which all collected data in blocks are chained together in an immutable, consentaneous, and encrypted manner [11]. Particularly, the information exchange between electronic medical records (EMRs), electronic health records (EHRs), and personal health records (PHRs) can be securely established. It has been found that blockchain technology has a great potential to protect the sensitive and confidential data of the healthcare industry, as well as to create a reliable data exchange mechanism between IoT-based healthcare devices. Recent years have seen a growing tendency to investigate the possibility of integrating blockchains and the IoT within healthcare management [12]. A decentralised and privacy-preserving healthcare management can be established to overcome the challenges raised by simple IoT-based healthcare solutions. Consequently, we will consider this integration so as to formulate secure and privacy-preserving data transmission for long-term care management, while simultaneously extracting the collected data in order to achieve nursing staffing optimisation.

### 2.2. Factors Affecting Nursing Staffing Optimisation

Personnel planning is central to an organisation's strategic and human resources planning process [13]. Numerous studies have investigated personnel planning in healthcare organisations specifically, such as nurse and doctor scheduling in hospitals [14, 15] and nursing staffing level planning and scheduling in nursing homes [16, 17]. Service schedule modelling and nursing staff assignment have been studied widely in the context of healthcare settings, such as medical centres [18] and home-care companies [19]. However, it has been found that the determination of the appropriate nurse staffing level in nursing homes is consistently hindered by budgetary constraints, talent shortages, and a lack of empirical evidence to guide and make adequate staffing decisions. Instead of acute treatments in hospitals, long-term care services are gradually promoted as addressing society's ageing population—where nursing homes are regarded as the essential long-term care facilities in any community. Therefore, scholarly attention to nursing staff optimisation has risen considerably in recent years. The nursing workforce planning has many characteristics, such as noninventoriable services and time-varying demands, thus making it far more complicated than traditional workforce planning issues. To meet peak and fluctuating demands, some researchers have proposed floating nurse pools, on-the-job training, and cross-training to increase staff flexibility [15, 20]. Nasiri and Rahvar [21] developed a nurse scheduling model which considered nurse preferences and consecutive shifts. Although the optimal schedule would satisfy both the hospital and staff's preferences, staff-task flexibility referring to the allocation of qualified staff to specific professional tasks has been insufficiently considered. In the context of nursing homes, residents generally require nursing staff assistance to complete a number of daily activities and all-day-round nursing and medical cares. In general, there are two staff assignment models: consistent and rotational assignment [22]. The former schedules/assigns staff to the same resident on most shifts, thereby allowing for close bonds to form between nursing staff and residents. Conversely, the latter model distributes the care burden among all available staff such that the flexibility of care services can be greatly enhanced. Furthermore, residents' need for care is one of the most important factors affecting nursing workforce management [23]. Some studies have investigated the relationship between residents' characteristics and the nursing staffing level [24, 25]. Their findings are consistent with previous studies in which staffing hours and staffing levels were positively correlated with the resident case-mix in nursing homes.

### 2.3. Existing Approaches to Staffing Optimisation

Among limited research studies on staffing management formation in nursing homes, some optimisation problems were established at the task scheduling level [26], the nurse assignment level [27], an integration of routing and scheduling levels [28], and an integration modelling of nursing staff demand and scheduling [29]. Regarding the healthcare staff demand modelling problem, Greuningen et al. [30] reviewed and evaluated the Dutch simulation model which has now become an accepted instrument for estimating the required supply of health professionals in the Netherlands on a regular basis. On the other hand, Maass et al. [31] proposed the stochastic programming approach to consider a homogeneous workforce and constant staffing levels in hospital settings and with a limited capability to plan from a resident case-mix, skill-mix, or skill substitution perspective. As staffing optimisation is generally regarded as an NP-hard problem [32, 33], there is no efficient exact algorithm to solve the problem of realistic size under polynomial time, thereby resulting in a heavy computational burden for the optimisation process. Typically, a daily staffing optimisation problem is to minimise the number of staff members to finish a certain number of operations, as in equation (1), where *i* and *j* denote staff index and operation-hour index, respectively [34]. Such an integer programming model is constrained to required time in man-hour for designated operations and the binary integrality of the decision variable *x*_*ij*_.

(1) $$\begin{array}{c} \sum_{i=1}^{I}\sum_{j=1}^{24}x_{ij}. \end{array}$$

Therefore, it has become common practice to obtain near-optimal solutions for NP-hard staffing optimisation problems using evolutionary and heuristic methods [35]. In real-life situations, management tends to prefer efficient and reliable approaches to obtain optimal solutions, thus giving rise to evolutionary optimisation techniques over exact algorithms. A genetic algorithm (GA) is a meta-heuristic technique widely used for solving NP-hard optimisation problems to obtain optimal, or near-optimal, solutions [36]. Thus, a GA can be considered a reasonable tool to resolve the NP-hard nursing staffing optimisation problem (NSOP) within a short computational time while maintaining the quality of an optimal solution. Several studies have successfully applied GA-based methods within staff scheduling and healthcare service demand forecasting [37, 38]. In light of the above, we consider a GA-based approach to be highly suitable for our research aims and proposed system framework.

## 3. Design of a Blockchain-IOT-Driven System for Nursing Workforce Planning

This section proposes a blockchain-IoT-driven system for nursing workforce planning (BIoT-NWP), where blockchains and the IoT are used to build an effective data acquisition system from the elderly and nursing homes, and the corresponding optimisation problem is embedded to allocate optimal workforce performance for routine nursing care services. With the use of blockchain-IoT technology, parameters, such as service requirements, nursing tasks, and residents' characteristics, are collected and recorded in a secure and reliable manner to obtain the optimal nursing staffing solution.

### 3.1. Blockchain-IoT-Driven System Architecture

To facilitate workforce planning, the blockchain-IoT-driven system is developed to structure the data acquisition process from the elderly and nursing staff to provide the decision-making functionality of nursing staffing.  Figure 2 presents the layered architecture of the BIoT-NWP, containing perception, mist, fog, decentralisation, cloud, and application layers—all of which consider the blockchain and IoHT paradigms [10, 12, 39]. Due to the current severe situation of COVID-19 (COVID-19) pandemic, more and more research studies explored system-wide solutions to enhance the quality of care, while the risk management on personal health can be maintained at an appropriate level [40]. An effective healthcare system built from the IoT technology is an active research area [41]. Apart from understanding the healthcare scenarios and requirements, the development of the blockchain-IoT system architecture may also consider the typical taxonomy and protocols for real-time data exchange [42]. More importantly, secure access control on IoT devices plays an essential role to manage physical nodes and devices in the IoT-driven system [43], which can be further enhanced by incorporating the blockchain technology to formulate the decentralised access control. The system authentication and authorisation can be effectively established for smart city applications, including healthcare management.

#### 3.1.1. Perception Layer

The perception layer specifies the “things” to be interconnected to the digital world. To achieve the goal of nursing workforce planning, the customised care plans of elderly residents in nursing homes must be considered. The care plans contain long-term care information pertaining to caring needs, service plans, goals, and review processes, which are digitalised and accessed via tablets. Through the tablets' digital platform, the nursing staff can view and perform a list of nursing tasks, while various health monitoring devices are connected to assist such routine care services as monitoring vital signs and body temperature, as well as administering medicine. Nursing staff are afforded greater privileges and access within the platform than the elderly so as to create and modify the care services. Overall, the long-term care information platform collects the requirements and customisations from the elderly, while the nursing staff can use these to accomplish their required daily tasks.

#### 3.1.2. Mist Layer

The mist layer refers to the edge of the network fabric, which includes sensors and actuator controllers. Typically, this performs basic rule-based preprocessing of the sensor data, such as data aggregation, fusion, and filtering. The edge nodes (e.g., routers) are located in the wards to form a number of mist networks, to which the data from the digital platform are transmitted. Since edge nodes provide limited resources (e.g., power, memory, and communication bandwidth), a reasonable assignment of sensor and edge nodes is required. Particular to the power consumption, the power of communication—which is approximately five times that of computing power—tends to be eliminated.

#### 3.1.3. Fog Layer

Rather than solely relying on cloud-based mechanisms, the fog layer provides the high responsiveness and minimal latency of IoT solutions. A number of private clouds (in accordance with the number of nursing homes in the network) are established to provide various processing and analytics functions, such as data filtering, data compression, data analytics, short-term data storage, and data fusion. Computing resources and application services are placed closer to the edge so as to eliminate disposable load on the cloud and backbone bandwidth, resulting in the IoT system's reduced latency. Due to the fog layer's decentralised architectural pattern, there is room to further enhance the system security and reliability through applying decentralisation technologies, such as blockchains. From the nursing homes' perspectives, a set of service requirements and time-specific tasks can be stored in the private clouds in a structured manner.

#### 3.1.4. Decentralisation Layer

In view of facilitating transparency and interoperability between an organisation's various nursing homes, we propose a permissioned blockchain to consolidate service requirements and tasks such that a chain of records about activities can be established. Subsequently, the trends of service requirements and tasks can be effectively inspected under the blockchain mechanism. Considering the organisation structure in nursing homes, all nursing staff are directed by nursing home managers who are responsible for approving and mining the data to the blockchain. As shown in Figure 3, these manages can assign appropriate privilege on authorised nodes. Malicious and abnormal nodes can be effectively filtered from the permissioned blockchain. Additionally, the chain validation—including the consistency of hash and previous hash values and the longest-chain rule—is conducted to maintain the data's accuracy and reliability. Once the data are mined and validated in the blockchain, all nursing home nodes are then synchronised to obtain the global set of service requirements and tasks. Simply put, the data are decentralised in the permissioned peer-to-peer network to ensure the system's security and trustworthiness.

#### 3.1.5. Cloud Layer

Given that the blockchain avoids storing large volumes of datasets, the blockchain constructs the data chain of the associated identities (IDs) of service requirements and tasks. Conversely, the cloud layer is essential for storing tenured and permanent information of the service requirements and tasks, such as task details, pictures, and standard operating procedures. Other than the above information, inactive and completed blockchains are stored in the cloud for long-term storage, a procedure known as blockchain vaporisation. Further to long-term data storage and load balancing, the cloud database also includes advanced machine learning models and big data analytics processing engines for effective data analysis. All the data managed in the cloud and blockchian are used to determine the optimal nursing staffing level.

#### 3.1.6. Application Layer

In the application layer, the nursing workforce planning is considered as the core application of the proposed system, where the corresponding objective and constraints are defined to achieve the optimal nursing staffing solution with the application of the GA. With the help of blockchain, mist, fog, and cloud computing, the trend of nursing services can be investigated for prospecting the effective workforce planning in the next rostering period. The nursing staff can be effectively allocated to provide the maximum QoC at the lowest costs.

### 3.2. Preliminaries of the Nursing Staffing Optimisation Problem

Regarding the application layer of the BIoT-NWP, an NSOP is considered present when a set of healthcare services (or tasks) required by a set of residents must be completed by a set of available nurses. Each nurse belongs to a specific service category based on their own qualifications, skills, and experience. Residents have their own healthcare needs when living in nursing homes. In order to effectively manage the nursing staff, the goal of this optimisation is to determine an optimal staffing level in shifts with fixed start and end times for the roster creation. Prior to the planning stage, the nursing home manager uses the BIoT environment to collect residents' service requirements and the particulars of the nursing staff, such as their categories and monthly salaries. Residents can thus be nursed by designated staff, provided that the nurse fulfils the healthcare task's legal requirements (skill substitution). Instilling skill substitution without creating a homogeneous workforce provides staff-task flexibility and practical requirements. Consequently, a nursing home manager is responsible for assigning nursing staff to shifts who perform (at least) a set of healthcare tasks. There are two main types of residential care routinely provided by nursing staff, namely, direct and indirect care. Direct care refers to the amount of time nursing staff spend with residents, while indirect care is the time spent on other nursing tasks, such as documentation and reviews for residents' ICPs. Therefore, we propose formulating the model by considering both direct and indirect care.

The constraints of the proposed model can be divided into two aspects, namely, hard and soft constraints. The former must be satisfied at all times in order to generate a feasible and optimal nursing staffing plan [29]. The following elaborates the suggested hard constraints in the proposed model:

- *Restrictions on Service Requirements from Legislation and Service Agreements*. The legislation and service agreement on service and staffing requirements must be met.
- *Restrictions on Working Hours and Breaks from the Legislation and Employment Contracts*. Both contracts and legislation concern the maximum length of continuous work within a day, the maximum number of continuous days worked, the minimum length of continuous rest between shifts, as well as other limits—all of which must be met.
- *Days Off and Leave Requested by Nursing Staff*. Days off and leave are considered a hard constraint that ensures that no staff member is assigned a shift on a day-off or on leave.
- *Rest Period between Shifts*. The work schedule of nursing staff is split into a number of shifts throughout the day. A rest period is essentially provided between two shifts.
- Soft constraints, however, are desired but not compulsory in the optimisation model and can be violated if necessary. The following elaborates a suggested soft constraint in the proposed model:
- *Maximum Amount of Overtime*. The legislation and contracts on the maximum length of overtime within a day is given. Since overtime creates pressure on frontline nursing staff and might increase the staff turnover rate, less overtime for each nursing staff is desirable.

### 3.3. Model of the Nursing Staffing Optimisation Problem

To formulate the optimisation model of the NSOP, the notations are defined in Table 1 with some sets/variables referred to a previous study [29].

The proposed model contains two sets of binary variables to monitor the staffing level and staff assignment. The binary variable *A*_*ijm*_ determines whether a regular staff member *j* ∈ *D*_*i*_^*t*^ ∪ *D*_*i*_^″^ of category *i* ∈ *C* is working in shift *m* ∈ *S* where *D*_*i*_ is the set of nursing staff of category *i*, *D*_*i*_′ is the set of potential nursing staff of category *i* to be hired, *C* is the set of nursing staff categories, and *S* is the set of shifts in the planning horizon. Similarly, the binary variable *B*_*ijm*_^*t*^ determines whether a temporary staff member *j* ∈ *D*_*i*_ ∪ *D*_*i*_′ of category *i* ∈ *C* is working in shift *m* ∈ *S*. Further to the staffing level, the proposed model contains two sets of nonnegative integral variables to document the working hours of nursing staff across the various shifts. The integral variable *T*_*ijm*_^*ot*^ determines the hours of overtime conducted by regular nursing staff *j* ∈ *D*_*i*_^*t*^ ∪ *D*_*i*_^″^ of category *i* ∈ *C* in shift *m* ∈ *S*. The integral variable *T*_*ijm*_^*t*^ determines the working hours of temporary nursing staff *j* ∈ *D*_*i*_ ∪ *D*_*i*_′ of category *i* ∈ *C* in shift *m* ∈ *S*. The ultimate objective of the proposed model is to plan for the number of staff required in each category to fulfil all of the residents' requirements with a minimum total monthly staffing cost (*Z*). The optimisation model is, therefore, expressed as in equation (2), which is measured in dollar values. Various costs related to manpower, such as those associated with the hiring and firing of staff, are considered and summed, allowing the staffing plan to be evaluated. As the objective function (2) does not consider the preferences of individual staff or the biases of the nursing home manager, the objective function consequently (and naturally) balances the workload of the available nursing staff.

(2) $$\begin{array}{c} \text{Min}.Z=\sum_{i\in c}\sum_{j\in D_{i}UD_{i}^{\prime }}\left(X_{ij}S_{ij}+R_{ij}^{\text{otp}}\sum_{m\in S}T_{ijm}^{\text{ot}}\right)+\sum_{i\in C}\left(C_{i}^{h}N_{i}^{h}+C_{i}^{f}N_{i}^{f}+C_{i}^{t}T_{i}^{t}\right) \end{array}$$

where

(3) $$\begin{array}{c} T_{i}^{t}=\sum_{j\in D_{i}\cup D_{i}^{\prime }}\underset{m\in S}{\sum }T_{ijm}^{t},\;\forall i\in c, \end{array}$$

(4) $$\begin{array}{c} X_{\mathrm{ij}}=\left\{\begin{array}{cc} 1\text{,} & \text{if }\sum_{m\epsilon S}A_{\mathrm{ijm}}\geq 1,\\ \text{0,} & \text{Otherwise,} \end{array}\right.\;\forall i\in C,\;\forall j\in D_{i}\cup D_{i}^{\prime }, \end{array}$$

(5) $$\begin{array}{c} X_{ijq}=\left\{\begin{array}{cc} 1, & \text{if }\sum_{m\in S}X_{ijm}\geq 1,\\ 0, & \text{otherwise}, \end{array}\right.\;\forall i\in C,\;\forall j\in D_{i}\cup D_{i}^{\prime },\;\forall q\in Q^{\prime }, \end{array}$$

(6) $$\begin{array}{c} N_{i}^{h}=\sum_{j\in D_{i}\cup D_{i}^{\prime }}\underset{q\in Q^{\prime }}{\sum }\left\{X_{ijq}-X_{ij\left(q-1\right)}\right\},\;\text{if }X_{ijq}=1,\;\forall i\in C, \end{array}$$

(7) $$\begin{array}{c} N_{i}^{f}=\sum_{j\varepsilon D_{i}\cup D_{i}^{\prime }}\underset{q\in Q^{\prime }}{\sum }\left\{X_{\mathrm{ij}\left(q-1\right)}-X_{\mathrm{ijq}}\right\},\;\text{if }X_{\mathrm{ijq}}=0,\;\forall i\in C, \end{array}$$

(8) $$\begin{array}{c} T_{i}^{t}=\sum_{j\in D_{i}^{t}\cup D_{i}^{\prime \prime }}\sum_{m\epsilon S}T_{\mathrm{ijm}}^{t},\;\forall i\in C, \end{array}$$

subject to

(9) $$\begin{array}{c} \sum_{i\in C}\sum_{j\varepsilon D_{i}\cup D_{i}^{\prime }}\left(A_{\mathrm{ijm}}U+T_{\mathrm{ijm}}^{\mathrm{ot}}\right)+\sum_{i\in C}\sum_{j\varepsilon D_{i}D_{i}^{\prime }}B_{\mathrm{ijm}}^{t}\cdot T_{\mathrm{ijm}}^{t}\geq \sum_{i\in C}\sum_{k\in R}\sum_{l\in T}N_{\mathrm{kl}}T_{\mathrm{ikl}}Y_{\mathrm{klm}},\;\forall m\in S, \end{array}$$

(10) $$\begin{array}{c} U+T_{ijm}^{ot}\leq \left(U+T_{ijm}^{ot}\right)\cdot A_{ijm\;},\;\forall i\in C,\;\forall j\in D_{i}\cup D_{i}^{\prime },\;\forall m\in S, \end{array}$$

(11) $$\begin{array}{c} T_{ijm}^{t}\leq T_{ijm}^{t}\cdot B_{ijm}^{t},\;\forall i\in C,\;\forall j\in D_{i}^{t}\cup D_{i}^{\prime \prime },\forall m\in S, \end{array}$$

(12) $$\begin{array}{c} \sum_{m=\left\{1,22,43,64\right\}}^{m+20}A_{ijm}=X_{i}^{w,\max},\;\forall i\in C,\;\forall j\in D_{i}\cup D_{i}^{\prime }, \end{array}$$

(13) $$\begin{array}{c} 0\leq A_{ijm}+A_{ij\left(m+1\right)}\leq 1,\;\forall i\in C,\;\forall j\in D_{i}\cup D_{i}^{\prime },\;\forall m\in S, \end{array}$$

(14) $$\begin{array}{c} 0\leq B_{ijm}^{t}+B_{ij\left(m+1\right)}^{t}\leq 1,\;\forall i\in C,\;\forall j\in D_{i}^{t}\cup D_{i}^{\prime \prime },\;\forall m\in S, \end{array}$$

(15) $$\begin{array}{c} \sum_{m=\left\{1,\;4,7,\ldots ,85,\;88\right\}}^{m+2}A_{ijm}\leq 1,\;\forall i\in C,\;\forall j\in D_{i}\cup D_{i}^{\prime }, \end{array}$$

(16) $$\begin{array}{c} \sum_{m=\left\{1,\;4,7,\ldots ,85,\;88\right\}}^{m+2}B_{ijm}^{t}\leq 1,\;\forall i\in C,\;\forall j\in D_{i}^{t}\cup D_{i}^{\prime \prime }, \end{array}$$

(17) $$\begin{array}{c} 0\leq T_{ijm}^{ot}\leq O_{im}^{\max}\cdot A_{ijm},\;\forall i\in C,\;\forall j\in D_{i}\cup D_{i}^{\prime },\;\forall m\in S, \end{array}$$

(18) $$\begin{array}{c} 0\leq T_{ijm}^{t}\leq T_{i}^{\max}\cdot B_{ijm}^{t},\;\forall i\in C,\;\forall j\in D_{i}^{t}\cup D_{i}^{\prime \prime },\;\forall m\in S, \end{array}$$

(19) $$\begin{array}{c} X_{ijw}^{t}=\left\{\begin{array}{cc} 1, & \text{if }\sum_{m=1}^{84}B_{ijm}^{t}\geq 1,\\ 0, & \text{otherwise}, \end{array}\right.\;\forall i\in C,\;\forall j\in D_{i}\cup D_{i}^{\prime }, \end{array}$$

(20) $$\begin{array}{c} E_{ijw}^{t}=\sum_{m=\left\{1,22,\;43,\;64\right\}}^{m+20}T_{ijm}^{t}\;\leq T_{i}^{w,\max},\;\forall i\in C,\;\forall j\in D_{i}\cup D_{i}^{\prime },\forall w\in W^{\prime }, \end{array}$$

(21) $$\begin{array}{c} N_{iw}^{t}=\sum_{j\in D_{i}\cup D_{i}^{\prime }}X_{ijw}^{t},\;\forall i\in C,\;\forall w\in W^{\prime }, \end{array}$$

(22) $$\begin{array}{c} A_{ijm}\in \left\{0,\;1\right\},\;\forall i\in C,\;\forall j\in D_{i}\cup D_{i}^{\prime },\forall m\in S, \end{array}$$

(23) $$\begin{array}{c} B_{ijm}^{t}\in \left\{0,\;1\right\},\;\forall i\in C,\;\forall j\in D_{i}^{t}\cup D_{i}^{\prime \prime },\;\forall m\in S. \end{array}$$

Equations (3) to (8) define *T*_*i*_^*t*^,  *X*_*ij*_, *X*_*ijq*_,  *N*_*i*_^*h*^, *N*_*i*_^*f*^, and *T*_*i*_^*t*^, respectively, to support the formulation of the objective function. Equation (9) ensures that both the direct and indirect care demands of all residents (in staff hours) can be satisfied within each shift by either regular or temporary nursing staff, and all unserved staff hours cannot be stocked. The minimum estimated demand for resident care (in staff hours) during shift *m* was forecast based on three years of historical data. Moreover, we considered seasonal characteristics during the demand forecasting, as represented by ∑_*i*∈*C*_∑_*k*∈*R*_∑_*l*∈*T*_*N*_*kl*_*T*_*ikl*_*Y*_*klm*_. Constraint (10) limits the number of working hours for each selected regular nursing staff. If the regular nursing staff is not selected for the shift *m*, this constraint prohibits the model from assigning hours to this regular nursing staff in shift *m*. Similarly, Constraint (11) limits the number of working hours for each selected temporary nursing staff. If the temporary nursing staff is not selected for the shift *m*, this constraint prohibits the model from assigning hours to this temporary nursing staff in shift *m*. Equation (12) handles the number of shifts that a regular staff member should perform in every 7 consecutive days, which is equivalent to 7 days × 3 shifts per day, namely, a total of 21 shifts per week. We assumed there to be 4 weeks in every month, such that the total number of shifts per month is 84. This constraint also ensures that one day-off per week is assigned to each selected regular nursing staff. Temporary nursing staff can be hired when the residents' service demand level (in staff hours) cannot be satisfied by existing regular nursing staff within each shift and when hiring additional regular nursing staff is unfavourable. Equations (13) and (14) ensure that regular and temporary nursing staff, respectively, cannot undertake consecutive shifts. Equations (15) and (16) prohibit the model from assigning more than one shift per day (i.e., 3 shifts) on each selected regular and temporary nursing staff, respectively. In other words, the equations ensure that there shall be no split shift, comprising more than one period of duty in a day, to be scheduled. Equation (17) expresses the limitation imposed on regular nursing staff concerning the maximum number of overtime work (in hours) a regular nursing staff member can work per shift. Equation (18) limits the maximum number of working hours a temporary nursing staff who can work per shift. Equation (19) defines the relationship between *B*_*ijm*_^*t*^ and *X*_*ijw*_^*t*^. Specifically, when a temporary nursing staff is selected for any shift within twenty-one consecutive shifts (i.e., seven consecutive days), the temporary staff is counted in the workforce in that particular week. Equation (20) defines the relationship between *T*_*ijm*_^*t*^ and *E*_*ijw*_^*t*^ and expresses the limitation imposed on temporary staff concerning the maximum number of working hours that a temporary nursing staff can work per week. Hence, the weekly number of temporary nursing staff, for each category, to be hired is given by equation (21). Equations (22) and (23) define *A*_*ijm*_ and *B*_*ijm*_^*t*^ which are binary variables. Overall, the proposed model seeks to find an optimal level of nursing staff, hopefully with fewer overtime hours, with the lowest total monthly staffing cost.

## 4. Solution Algorithm

This optimisation problem is modelled in three-dimensional space of number of staff categories, number of staff members per category, and number of shifts, and therefore the computational complexity can be expressed as *O*(*I* × *D*_*i*_!×*S*). When the number of staff categories and number of shifts are predefined and fixed by the nursing homes, the computational complexity is at least *O*(*D*_*i*_!) to determine the optimal sequence of staff members per the category *i*. In order to effectively solve the proposed model with the NP-hard characteristics in a high run-time complexity environment, we selected the GA to formulate a customised solution algorithm to obtain an optimal (or near-to-optimal) solution. We applied a constructive heuristic approach to generate initial feasible solutions, while the GA was applied to improve the quality of solutions through iterations. The solution of the optimisation problem using the GA requires the corresponding individual representation for the decision variables *A*_*ijm*_, *B*_*ijm*_^*t*^, *T*_*ijm*_^*ot*^, and *T*_*ijm*_^*t*^. *A*_*ijm*_ and *B*_*ijm*_^*t*^ are expressed as binary variables, while *T*_*ijm*_^*ot*^ and *T*_*ijm*_^*t*^ are expressed as nonnegative integers. The length of the chromosome depends on the number of nursing staff categories (*i*), the number of staff within a category (*J*_*I*_), and the number of shifts (*M*). A chromosome is composed of 1+∑*J*_*I*_ sections, and there are (∑*J*_*I*_) × *M* units in the first section and *M* units in the remaining sections. The first section contains information as to whether the nursing staff is selected and assigned to a particular shift, i.e., counted in the workforce. The remaining sections contain information on the amount of overtime conducted by regular nursing staff in the shift, or information on the number of work hours for a temporary nurse in the shift. The binary variables *A*_*ijm*_ and *B*_*ijm*_^*t*^ are ordered by the shift *m*, nursing staff category *I*, and staff indicator *j*. The overtime and work hour variables are ordered by the shift *m*. As an example, the encoding scheme for one regular nursing staff category, one temporary nursing staff category, one member of staff in each category, and three shifts is as follows: [*A*_111_, *B*_111_^*t*^, *A*_112_, *B*_112_^*t*^, *A*_113_, *B*_113_^*t*^, *T*_111_^*ot*^, *T*_112_^*ot*^, *T*_113_^*ot*^, *T*_111_^*t*^, *T*_112_^*t*^, *T*_113_^*t*^].

Figure 4 shows the graphical illustration of the above example. For shift 1, information on the chromosome includes the following: regular nursing staff member 1 of Category 1 is on-duty (*A*_111_=1) with an overtime of 4 hours (*T*_111_^*ot*^ = 4). For shift 2, temporary staff member 1 of Category 1 is on-duty (*B*_112_^*t*^=1) with a working time of 6 hours (*T*_112_^*t*^=6). For shift 3, neither staff member 1 nor 2 of Category 1 is on-duty (*A*_113_=*B*_113_^*t*^=0), and thus no working hours or overtime is allowed (*T*_113_^*ot*^=*T*_113_^*t*^=0). The initial population consists of the solutions from the constructive heuristic method. The constructive heuristic approach begins with an empty workforce plan. A feasible workforce plan is obtained by adding or removing particular staff and work hours from the initial plan until the hard constraints are met. In order to obtain the problem's optimal solution, the genetic operations, including selection, crossover, and mutation, must be performed to update the solution iteratively [44]. Consequently, the optimal nursing staffing plan with the lowest costs can be established.

## 5. Case Study and Analysis

This section will provide a case study and analysis in order for us to verify the feasibility and effectiveness of the proposed system in a nursing home environment. We investigated a nursing home in Hong Kong for the deployment of the proposed BIoT system and the solution of a real-world NSOP. Consulting the nursing home managers enabled us to identify and summarise certain existing challenges:

- The monthly staffing level required is estimated by the nursing home managers based on intuition and past experience
- The schedule is produced manually once every two weeks, thus making a digital solution desirable
- The average time taken for producing a biweekly schedule is at least two hours, which is not a value-added activity
- Workforce planning problems, such as balancing the staff load, spreading the nursing staff across shifts, and fulfilling legal requirements, occur frequently

The proposed system seemed likely to overcome the above challenges, and therefore the nursing home company was invited to implement it. The entire implementation was divided into three parts, namely, (i) BIoT system deployment, (ii) parameter settings of the NSOP, and (iii) numerical results and discussion.

### 5.1. Blockchain-IoT System Deployment

Figure 5 shows the deployment of the long-term care platform for residents and care workers, where the list of tasks with designated start and end periods is displayed. The individual tablets were assigned to the residents and installed next to their berths. The care workers' ID cards were used to activate the dashboard to view all the required care tasks for specific residents. The workers could record their care services upon completion. In the wards, a full Wi-Fi coverage was provided such that the long-term care platform data could be effectively transmitted to the private cloud controlled by nursing home managers via an edge device (router). The care service data were collected to construct a data chain regarding the nursing home's service requirements.

Other than the service requirements update, other data (e.g., documentations) are stored long-term by cloud computing. In other words, the proposed system suggests a hybrid design of blockchain and cloud computing. Overall, the parameters regarding care services, residents, and care workers are organised so as to most effectively optimise nursing staffing.

Table 2, describes six aspects of the blockchain: data in blocks, consensus algorithm, encryption method, validators, data collection nodes, and expected network size. In the blockchain, each data block contains hash value, previous hash value, data, timestamp, and nonce (an arbitrary number used in a cryptographic communication). Moreover, the hash values in data blocks are generated by using the secure hash algorithm 256 (SHA256), such that the hash values are in 256-bit (or 32 bytes). The entire block building process is illustrated in Figure 6 where the data of service tasks are stored in a tree structure to manage completed and pending activities. To further enhance the system security of the data exchange, asymmetric encryption was applied to encrypt the data to the cipher text by using public and private key pairs, where public keys were referred to the addresses in the P2P network. Since the proposed system requires the construction of a consortium blockchain among various branches of nursing homes, we considered the use of the voting-based consensus algorithm, Istanbul Byzantine Fault Tolerance (IBFT). One of the validators (in this case nursing home managers) is selected as the proposer to construct a block in the blockchain when a two-thirds majority of validators declares the new block to be valid. In order to maintain the blockchain's stability, the expected network size contains (3*F* + 1) nodes, where *F* refers to the estimated number of malicious nodes. Simply put, the proposed blockchain mechanism is able to tolerate at most *F* malicious nodes which attempt to dominate the blockchain.

### 5.2. Implementation Details of the NSOP

Regarding the implementation details, the model parameters for the case study are defined as shown in Table 3, where there are five nursing staff members in the Category 1, two nursing staff members in the Category 2, and two nursing staff members in the Category 3 working in the nursing home. The baseline of the total monthly staffing cost is HK$319,500. Also, no temporary staff have been employed, and the regular nurses occasionally work overtime in order to complete all of the care tasks within the shifts. According to the observation, it is assumed that (i) the marginal cost associated with employment and layoff of regular staff in nursing homes remains constant and equals the monthly salary of the nursing staff; (ii) regular nurses' monthly salaries are based on their staff grade (termed “nursing staff category” in the proposed model), subject to a minimum set at the midpoint, which are used when undertaking nursing staffing optimisation; and (iii) elderly patients staying in nursing homes are identical. The service time of individual healthcare tasks performed in a particular shift (*N*_*k*_ × *T*_*ikl*_ × *Y*_*klm*_) is named as “total required service time (in minutes).” Based on the above model parameters and assumptions, the NSOP is then solved to evaluate the total monthly staffing cost, which is the value of the objective function and the key evaluation parameter. In addition, the entire optimisation is conducted in MATLAB® R2019a in the 64-bit operating system (Windows 10) of i7-6770HQ CPU @2.60 GHz and 32 GB installed memory.

Furthermore, the GA parameters, namely, crossover rate (CR), mutation rate (MR), and population size (PS), were selected based on preliminary experiments to obtain the minimised fitness value in the NSOP. We considered 60 sets of combinations within the experiments, where the average fitness values (*Z*) were obtained by considering 20 independent runs (see Table 4). Moreover, the optimisation problem was solved in the Java environment, where the objective function and constraints were programmed. We found that the crossover rate of 1, the mutation rate of 0.1, and the 500 population size chromosomes provide the solution with the lowest total monthly staffing cost. Therefore, the parameter settings in using GA can be determined to solve the optimisation problem.

### 5.3. Numerical Results and Discussion

Given that the implementation details have been determined, the resulting nursing staffing optimisation computed by using the GA is analysed in this section by considering the following performance metrics. Firstly, percentage of the fulfilment of care demand by using either homogeneous or heterogeneous workforce is considered. Secondly, the monthly staffing cost (i) with or without considering heterogeneous workforce and (ii) with or without temporary staff is evaluated. According to the results of the above analyses, an optimal nursing staffing strategy can be formulated to determine the optimal nursing staff schedule in nursing homes.

#### 5.3.1. Percentage of Completed Healthcare Tasks

The percentage of completed healthcare tasks, both with and without the consideration of a heterogeneous workforce and skill substitution, is plotted in Figure 7. “Category 1” refers to a homogeneous workforce consisting of only Category 1 nursing staff—the same is true, respectively, of “Category 2” and “Category 3.” “All categories” refer to a heterogeneous workforce consisting of nursing staff of all categories and the absence of skill substitution. “Shift A” refers to the daytime shift, “Shift P” to the evening shift, and “Shift N” to the overnight shift. The results show that all care demands of the residents were fully satisfied when a heterogeneous workforce or a homogeneous workforce consisting of Category 3 nursing staff was employed and considered during the nursing workforce planning. However, it should be noted that some of the healthcare tasks could only be provided by the Category 3 nurses, meaning that homogeneous Category 1 and 2 workforces were unable to satisfy all of the residents' care demands.

#### 5.3.2. Total Monthly Staffing Cost When Using Heterogeneous versus Homogeneous Workforces

To illustrate the cost-effectiveness of a heterogeneous workforce while satisfying all care demands, we applied the GA to solve the cases of the homogeneous Category 3 workforce and a heterogeneous workforce. The comparison results obtained regarding the total monthly staff cost for these cases are shown in Figure 8. The results show that, in all of the 20 independent runs, using a heterogeneous workforce can achieve a lower total monthly staffing cost than using a homogeneous one. This fully validates the cost-effectiveness of our suggestion to apply heterogeneous workforces and skill substitution for nursing workforce planning.

#### 5.3.3. Total Monthly Staffing Cost with/without Temporary Staff

We also argue that the hiring of temporary nursing staff can enhance employment flexibility and cost-effectiveness. To illustrate cost-effectiveness, we contrasted the current situation (i.e., no temporary nursing staff having been employed and occasional need for regular nurses to work overtime) with the case of temporary nurses having been employed together with regular nurses working overtime. The comparison results regarding the total monthly staffing costs for these two cases are shown in Figure 9. “OT available, TEMP unavailable” refers to the current situation, while “OT & TEMP available” refers to the second case. The results show that the current situation, while being able to satisfy the residents' care demands, results in a higher total monthly staffing cost. Our proposed case, namely, hiring temporary staff, can achieve lower total staffing costs in all the 20 independent runs, thereby fully validating the cost-effectiveness of our approach.

#### 5.3.4. Total Monthly Staffing Cost: A Heterogeneous Workforce with Temporary Nursing Staff

From the results of Sections 5.3.1to 5.3.3, we can see the cost-effective nature of introducing temporary nursing staff, as well as considering heterogeneous workforces and skill substitution during nursing workforce planning. The nursing staff demand and the total monthly staffing costs for the case of a heterogeneous workforce together with temporary nursing staff and regular nurses working overtime are shown in Table 5. Upon inspection, we can see that the lowest and average total monthly staffing costs obtained from the proposed model are HK$270,340 and HK$276,442, respectively. In other words, they are equivalent to a 15.39% and 13.48% reduction of total monthly staffing costs when compared with the model based on the nursing home manager's perceived experience. As expected, there are significant decreases in the staffing levels of regular nurses, along with significant increases in the staffing levels of their temporary counterparts. These results indicate that when the residents' service demand levels (in staff hours) are high and fluctuate, the recruitment of temporary nursing staff tends to be more financially favourable over maintaining consistently high regular staffing levels for all work shifts. This reduction in monthly staffing costs could be explained by there being a sufficient supply of the required skills with more flexible staff hours.

Another finding is that a negative level change of regular nursing staff was significant for Category 1 nurses (i.e., the lowest nursing grade). This is predominant because residents can be nursed by various types of nursing staff provided that they fulfil the healthcare task's legal requirement of labour skills (skill substitution), and all of the care demands are suitably satisfied. Consequently, the proposed model tends to more effectively utilise regular nursing staff with higher monthly salaries (i.e., those in Category 3) as often as possible so as to ensure satisfying every care demand while simultaneously avoiding the unnecessary hiring of regular nursing staff from Category 1, who are incapable of fully satisfying care demands independently. Instead, the proposed model suggests recruiting temporary staff from Category 3. In other words, the results show that a mixed level of various nursing categories significantly impacts the total monthly staffing cost. This practice is becoming increasingly common in the healthcare industry in that the use of lower nurse grades, or support staff (e.g., patient care assistants), can effectively apportion simple clinical tasks and allay the nursing shortage.

### 5.4. Discussion on the BIoT-NWP

To address the resource shortage problem in nursing homes, the proposed system, namely, BIoT-NWP, considering the NSOP facilitates care monitoring and nursing staff optimisation. Compared with typical staff scheduling optimisation, this study presents an integrated approach to interconnect elderly care needs and requirements on a blockchain-IoT platform, where caregivers are effective to control and monitor the care services provided to the elderly. In addition, this platform collects a full list of care needs and requirements in an integrated manner, which can be utilised to schedule the nursing staff. This study can be seen as a milestone to digitalise the operations management in nursing homes. Regarding the practical implications, this study enhances the care services provided to the elderly by monitoring care needs and assigning optimal nursing staff in routine operations, and therefore the balance between quality of care and costs incurred in care services is struck. In other words, minimal cost on nursing staff scheduling in nursing homes can be determined, while all designated care needs and requirements can be fulfilled, resulting in improved quality of care. Besides, overlooking elderly's needs and requirements can be effectively prevented by means of the proposed blockchain-IoT solution. Overall, a track record about uncompleted and completed care services in nursing homes is maintained in an immutable and secure manner. On the other hand, the proposed system which can be regarded as a multidisciplinary study also contributes to the field of geriatric care management by integrating the blockchain, IoT, and optimisation problem, in which care service monitoring and nursing staff optimisation can be formulated accordingly. The practicality of the nursing staff optimisation can be further improved through incorporating the blockchain-IoT technology for effective data acquisition.

With the adoption of BIoT, the routine operations of nursing care are revamped to facilitate real-time health monitoring, care service control, and workforce planning, and therefore the operational flows and processes are changed accordingly. Although the advantages of using BIoT technologies can be leveraged in this study, the complexity of learning and using new technologies should be considered. Differing to the previous care services, the nursing staff is required to access the care service details and schedule through the smart devices, where some of them might resist the changes. Therefore, training sessions and workshops to explain the functions and advantages of the proposed approach are necessary. Also, additional technicians are needed to assist the nursing staff in the state of transition. Moreover, the overhead of adopting the proposed approach is subject to costs of smart devices (i.e., tablets and sensors), BIoT development, deployment of the NSOP, system evaluation, and maintenance. Referring to the trial run presented in the case study, the expected and actual overhead cost in total is about HK$350,000 and HK$380,000, respectively. Also, the total monthly staffing cost obtained by using the proposed approach is the activity driver to the overhead cost, such that the overhead rate of the proposed approach is $380,000/$276,442=1.37. In other words, the nursing home pays $1.37 in overhead cost for every staffing cost.

## 6. Concluding Remarks

In light of the global ageing population and worldwide challenge of a severe talent shortage in nursing homes, nursing workforce planning for enhancing the capacity of nursing homes and improving their working environment is more significant than ever before. In this study, the IoT-based long-term care information platform was designed to manage the ICPs of elderly residents, thereby providing care workers with a list of services to be performed. We integrated a blockchain mechanism in the above platform so as to decentralise the caring needs of nursing home networks, where the records of requested and completed care services can be chained in a secure and reliable manner. Regarding the nursing staffing optimisation based on the collected data, this study has actively considered the critical factors related to the care demand of residents, such as resident case-mix, staff-task flexibility, facilitation by adopting a heterogeneous workforce, hiring temporary nursing staff, and allowing for skill substitution. A mixed-integer programming (MIP)-based optimisation model is thus developed for staffing in nursing homes based on legislation, operational guidelines, and contracts with the nursing staff. The contribution of this study can be presented in two facets: firstly, the innovative synergistic integration of blockchain and the IoT facilitates operational research into nursing staffing; secondly, the proposed nursing staffing optimisation incorporates multiple essential factors as integral components of nursing homes so as to most effectively formulate a nursing workforce planning strategy to capitalise on workforces. For the future work, it is suggested that the proposed system can be further extended to other healthcare and residential care facilities, such as care homes, aged homes, and hospital to provide reliable health information recording platform and determine the optimal nursing staffing strategy. Additional objective functions, rather than monthly staffing cost, can be considered to strike a balance on multiple conflicting objectives, for example, quality of care, environmental impact, and operational costs. In so doing, the strategic and operational conflicts on nursing staff optimisation can be comprehensively resolved.

## Figures and Tables

**Figure 1:** Illustration of nursing home structure for staffing optimisation.

**Figure 2:** Layered architecture of the BIoT-NWP.

**Figure 3:** Graphical illustration of the blockchain mechanism in nursing homes.

**Figure 4:** An example for illustrating the encoded chromosome.

**Figure 5:** Deployment illustration of the long-term care platform.

**Figure 6:** Graphical illustration of the block building process.

**Figure 7:** Percentage of care demands of satisfied residents.

**Figure 8:** Total monthly staffing costs of using heterogeneous and homogeneous workforces.

**Figure 9:** Total monthly staffing costs with/without temporary nursing staff.

**Table 1:** Notations of the optimisation model of the NSOP.

Set/variable	Description
*C*	Set of nursing staff categories, *C* = {1, 2,…, *I*}
*D*_*i*_	Set of nursing staff in a particular category *i*, *D*_*i*_ = {1, 2,…, *J*_*i*_} where *J*_*i*_ is the given initial number of nursing staff of category *i*
*D*_*i*_^*t*^	Set of temporary nursing staff in a particular staff category *i*, *D*_*i*_^*t*^ = {1, 2,…, *J*_*i*_^*t*^} where *J*_*i*_^*t*^ is the given initial number of temporary nursing staff of category *i*
*D*_*i*_′	Set of potential nursing staff in a particular category *i* to be hired, *D*_*i*_′ = {*J*_*i*_+1, *J*_*i*_+2,…, *J*_*i*_+*J*_*i*_′} where *J*_*i*_′ is the given maximum permissible nursing staff of category *i* to be hired
*D*_*i*_^″^	Set of potential temporary nursing staff in a particular staff category *i* to be hired, *D*_*i*_^'′^ = {*J*_*i*_^*t*^+1, *J*_*i*_^*t*^+2,…, *J*_*i*_^*t*^+*J*_*i*_^″^} where *J*_*i*_^″^ is the given maximum allowable temporary nursing staff of category *i* to be hired
*R*	Set of resident types, *R* = {1, 2,…, *K*}. *S* set of shifts (in the planning horizon of 1 month), *S* = {1, 2,…, M}. *T* set of nursing tasks, *T* = {1, 2,…, *L*}
*P*_*i*_	Set of healthcare tasks that nursing staff of category *i* is qualified to perform, *P*_*i*_ = {1, 2,…, *L*_*i*_}
*W′*	Set of weeks (in a planning horizon), *W'* = {1, 2,…, *W*}
*Q′*	Set of month (in the planning horizon of 1 month), *Q*' = {1, 2,…, *Q*}
*T*_*i*_^max^	The upper limit of working hours per shift for a temporary staff of category *i*
*T*_*i*_^*w*,max^	The upper limit of working hours per week for temporary nursing staff of category *i*
*S*_*ij*_	Monthly salary of the *j*^th^ regular nursing staff of category *i*
*R*_ij_^otp^	Hourly wage of overtime for the *j*^*th*^ regular nursing staff of category *i*
*C*_*i*_^*h*^	Cost of hiring a regular nursing staff member of category *i*
*C*_*i*_^*f*^	Cost of having a regular nursing staff member of category *i* leaving the workforce
*C*_*i*_^*t*^	Hourly wage of temporary nursing staff of category *i*
*N*_*kl*_	Number of type *k* residents requiring the *l*^th^ healthcare task
*T*_*ikl*_	Service time (in minutes) of the *l*^th^ healthcare task for type *k* resident per shift if it is provided by nursing staff of category *i*
*Y*_*klm*_	1 if the *l*^th^ healthcare task is needed for type *k* resident in shift *m*; otherwise, 0
*X*_*i*_^*w*,max^	The upper limit of shifts a nurse of category *i* can undertake in every 7 consecutive days
*O*_im_^max^	The upper limit of overtime for a regular nurse of category *i* in shift *m*
*U*	Standard working hour for all regular nursing staff per shift
*N*_*i*_^*h*^	Number of additional regular nursing staff of category *i* to be hired
*N*_*i*_^*f*^	Number of existing regular nursing staff of category *i* who left the workforce
*N*_*iw*_^*t*^	Number of temporary nursing staff of category *i* in week *w*
*X*_*ij*_	1 if the *j*^th^ regular nursing staff of category *i* is counted in the workforce; otherwise, 0
*X*_*ijq*_	1 if *j*^th^ nurse of category *i* is counted in workforce for month *q*; otherwise, 0
*T*_*ijm*_^*ot*^	Overtime (in hours) for the *j*^th^ regular nursing staff of category *i* in shift *m*
*T*_*i*_^*t*^	Total working hours of temporary nursing staff of category *i*
*A*_*ijm*_	1 if the *j*^th^ regular nursing staff of category *i* is on-duty in shift *m*; otherwise, 0
*B*_*ijm*_^*t*^	1 if the *j*^th^ temporary nursing staff of category *i* is on-duty in shift *m*; otherwise, 0
*T*_*ijm*_^*t*^	Working hours of the *j*^th^ temporary nursing staff of category *i* in shift *m*
*X*_*ijw*_^*t*^	1 if the *j*^th^ temporary nursing staff of category *i* is counted in the workforce in week *w*; otherwise, 0
*E*_*ijw*_^*t*^	Total working hours of the *j*^th^ temporary nursing staff of category *i* in week *w*

**Table 2:** Specification of the proposed blockchain mechanism.

Aspects of blockchain	Detail(s)
Data in blocks	Hash value, previous hash value, data, timestamp, and nonce
Consensus algorithm	Istanbul Byzantine Fault Tolerance (IBFT)
Encryption method	SHA256 and asymmetric encryption
Validators	Nursing home manager
Nodes of data collection	Individual tablet of the residents
Expected network size	≥3*F* + 1, where *F* refers to the estimated number of malicious nodes

**Table 3:** Model parameters of the case company for nursing staffing optimisation.

	Value
*Parameter*	
*C*	{1, 2, 3}
*D*_1_	{1, 2, ..., 15}
*D*_2_, *D*_3_	{1, 2, ..., 6}
*D*_1_^*t*^, *D*_2_^*t*^, *D*_3_^*t*^	{0}
*Q′*	{1}
*D*_1_′	{16, 17,…, 30}
*D*_2_′, *D*_3_′	{7, 8,…, 12}
*R*	{1}
*S*	{1, 2,…, 90}
*T*	{1, 2,…, 28}
*W′*	{1, 2, 3, 4}
*T*_1_^*w*,max^, *T*_2_^*w*,max^, *T*_3_^*w*,max^	14
*S*_1*j*_, *C*_1_^*h*^, *C*_1_^*f*^	$8,500
*S*_2*j*_, *C*_2_^*h*^, *C*_2_^*f*^	$12,000
*D*_1_^″^	{1, 2, ..., 15}
*T*_1_^max^, *T*_2_^max^, *T*_3_^max^	12
*S*_3*j*_, *C*_3_^*h*^, *C*_3_^*f*^	$20,000
*R*_1*j*_^*otp*^	130
*R*_2*j*_^*otp*^	180
*R*_3*j*_^*opt*^	230
*C*_1_^*t*^	130
*C*_2_^*t*^	180
*C*_3_^*t*^	230
*D*_2_^″^, *D*_3_^″^	{1, 2, ..., 6}
*T*_1_^*w*,max^, *T*_2_^*w*,max^, *T*_3_^*w*,max^	18
*N*_1_	53
*X*_1_^*w*,max^, *X*_2_^*w*,max^, *X*_3_^*w*,max^	6
*O*_1*m*_^max^, *O*_2*m*_^max^, *O*_3*m*_^max^	4
*U*	8

*Other information*	
Total service time (in minutes) required in shift 1, 4, 7,…, 82, 85, 88	1725
Total service time (in minutes) required in shift 2, 5, 8,…, 83, 86, 89	2355
Total service time (in minutes) required in shift 3, 6, 9,…, 84, 87, 90	1020
Total monthly staffing cost	$319, 500

**Table 4:** GA parameter settings and results from problem instances.

#	CR	MR	PS	*Z*
1	0.2	0.1	100	359167.5
2	0.2	0.1	300	342215
3	0.2	0.1	500	326090
4	0.2	0.2	100	349168
5	0.2	0.2	300	330458
6	0.2	0.2	500	331318
7	0.2	0.4	100	355022
8	0.2	0.4	300	322926
9	0.2	0.4	500	323452
10	0.2	0.6	100	349024
11	0.2	0.6	300	320508
12	0.2	0.6	500	314732.5
13	0.4	0.1	100	348692.5
14	0.4	0.1	300	330700
15	0.4	0.1	500	307064
16	0.4	0.2	100	336270
17	0.4	0.2	300	318356
18	0.4	0.2	500	306075.6
19	0.4	0.4	100	349052
20	0.4	0.4	300	316696
21	0.4	0.4	500	310492.5
22	0.4	0.6	100	355078
23	0.4	0.6	300	312770
24	0.4	0.6	500	303615
25	0.6	0.1	100	328502.5
26	0.6	0.1	300	305405
27	0.6	0.1	500	293784.4
28	0.6	0.2	100	333720
29	0.6	0.2	300	304138
30	0.6	0.2	500	297088
31	0.6	0.4	100	331968
32	0.6	0.4	300	309064
33	0.6	0.4	500	304075
34	0.6	0.6	100	337504
35	0.6	0.6	300	308486
36	0.6	0.6	500	302227.5
37	0.8	0.1	100	330810
38	0.8	0.1	300	302394
39	0.8	0.1	500	302164
40	0.8	0.2	100	318124
41	0.8	0.2	300	297856
42	0.8	0.2	500	297772
43	0.8	0.4	100	326342
44	0.8	0.4	300	296394
45	0.8	0.4	500	298035
46	0.8	0.6	100	333254
47	0.8	0.6	300	299238
48	0.8	0.6	500	299877.5
49	1.0	0.1	100	307922.5
50	1.0	0.1	300	300762
**51**	**1.0**	**0.1**	**500**	**286524**
52	1.0	0.2	100	325412
53	1.0	0.2	300	294498
54	1.0	0.2	500	294476
55	1.0	0.4	100	315132
56	1.0	0.4	300	294194
57	1.0	0.4	500	290332.5
58	1.0	0.6	100	314700
59	1.0	0.6	300	310074
60	1.0	0.6	500	289978.8

*Note.* The bold parameter settings represent that the minimal fitness value was obtained.

**Table 5:** Details of the obtained optimal solutions

Run	No. of Category 1 regular nursing staff required	No. of Category 2 regular nursing staff required	No. of Category 3 regular nursing staff required	Level change∗ for Category 1 regular nursing staff	Level change∗ for Category 2 regular nursing staff	Level change∗ for Category 3 regular nursing staff	No. of Category 1 temporary nursing staff required	No. of Category 2 temporary nursing staff required	No. of Category 3 temporary nursing staff required	Total monthly staffing cost (HK$)
1	2	6	5	−13	0	−1	6	4	1	275,000
2	3	6	6	−12	0	0	6	5	3	277,480
3	4	5	6	−11	−1	0	5	4	0	270,340
4	6	5	4	−9	−1	−2	5	4	0	274,080
5	5	4	5	−10	−2	−1	5	6	1	284,260
6	4	5	6	−11	−1	0	5	5	0	273,980
7	5	5	5	−10	−1	−1	5	5	2	284,540
8	6	4	5	−9	−2	−1	6	2	1	274,200
9	5	4	6	−10	−2	0	5	4	0	271,640
10	5	6	6	−10	0	0	5	3	0	273,140
11	6	5	5	−9	−1	−1	5	3	1	272,580
12	5	6	4	−10	0	−2	6	3	2	280,520
13	4	4	6	−11	−2	0	5	4	1	274,800
14	5	4	5	−10	−2	−1	6	6	0	281,860
15	6	5	4	−9	−1	−2	6	3	0	280,820
16	4	5	6	−11	−1	0	5	4	0	274,780
17	5	5	5	−10	−1	−1	4	4	0	279,080
18	4	4	6	−11	−2	0	6	1	1	272,400
19	6	5	4	−9	−1	−2	6	5	0	276,860
20	6	4	5	−9	−2	−1	6	4	0	276,480
									Average	276,442 (−13.48%)

^∗^For level change, a positive number refers to the additional regular nursing staff to be hired, while a negative number refers to the amount of existing regular nursing staff left the workforce.

## Data Availability

The data used to support this study are included within the article.
